RETRACTED

# Clinical Observation of General Anesthesia Combined with Spinal Anesthesia in Elderly Patients with Chronic Obstructive Pulmonary Disease

**DOI:** 10.1155/2022/9160145

**Published:** 2022-08-21

**Authors:** Jie Chen, Jing Wang, Xiaohui Duan, Fumin Ping, Aiming Zhang

**Affiliations:** Affiliated Hospital of Hebei Engineering University, Handan, 056002 Hebei, China

## Abstract

**Objective:**

This work is aimed at evaluating the efficacy and safety of general anesthesia (GA) combined with spinal anesthesia (SA) (GA+SA) in elderly patients with chronic obstructive pulmonary disease (COPD). *Methods and Material*. 50 elderly COPD patients were rolled randomly into a control group (simple GA) and observation group (GA+SA). The differences in operation time, postoperative recovery time (PRT), language expression time (LET), anesthetic dosage (AD), catheter extubation time (CET), respiratory circulation indicators (mean arterial pressure (MAP), heart rate (HR), SaO_2_, and PaO_2_), postoperative VRS score, pulmonary function (forced vital capacity (FVC)), forced expiratory volume in 1 s (FEV1)/FVC and forced expiratory flow (FEF 25%~75%), serum inflammatory factors (IL-6, IL-8, and TNF-*α*), Short Portable Mental Status Questionnaire (SPMSQ) score, and the incidence of respiratory system events were analyzed.

**Results:**

The results showed that the PRT, LET, AD, and CET of the observation group were all shorter (*P* < 0.05). The postoperative MAP, HR, SaO_2_, and PaO_2_ levels of patients who received GA+SA were much higher than those who received simple GA (*P* < 0.05). The postoperative VRS score of the observation group was better than that of the controls (*P* < 0.05). The postoperative pulmonary function of patients in the observation group was better compared with that in the control group (*P* < 0.05). The postoperative serum inflammatory factors in the observation group were lower in contrast to the patients who received simple GA (*P* < 0.05). The postoperative cognitive function SPMSQ score of patients who received GA+SA was lower compared with the score of patients who received simple GA (*P* < 0.05). However, the probability of respiratory system events in the observation group was lower (*P* < 0.05).

**Conclusion:**

In conclusion, GA+SA could significantly shorten the PRT and improve the recovery quality of elderly COPD patients. It can also reduce the postoperative inflammatory response and strengthen the pulmonary function and cognitive function. It also enhances the analgesic which is beneficial to patients' postoperative recovery. Therefore, GA+SA was a highly effective and safe anesthesia method for elderly patients with COPD, and it was worthy of clinical application.

RETRACTED

## 1. Introduction

Chronic obstructive pulmonary disease (COPD) is a common disease characterized by persistent respiratory symptoms and airway airflow limitation [1]. COPD in patients is a chronic inflammatory lung disease that causes blockage of airflow in the lungs. This may lead to difficulty in breathing, cough, and mucus (sputum) production. The factors that lead to such disease may include long-term exposure to irritating gases or particulate matter, mostly from exposure to cigarette smoke. People having COPD are more likely to suffer from heart disease, lung cancer, and a variety of other conditions [2]. The main clinical features of COPD are chronic cough, expectoration, chest tightness, shortness of breath, and dyspnea. Severe COPD patients also have problems such as weight loss and loss of appetite [3]. Clinical studies have confirmed that COPD patients have high mortality and morbidity rates, and it is one of the reasons for the increased mortality and morbidity of patients worldwide [4, 5]. With the deepening of population aging, the incidence of COPD also shows an increasing trend year by year. In addition, the elderly are the high-risk group for the COPD due to the reduced function of the immune system, the enlargement of the alveolar space, the reduction of the compliance of the lung tissue, the weakening of the respiratory muscle strength, the cough reflex, and the coexistence of multiple diseases and malnutrition [6, 7]. Although COPD is a progressive disease that gets worse over time, COPD is treatable. With proper management, most people with COPD can achieve good symptom control and quality of life, as well as reduced risk of other associated conditions. At present, surgery is the main method for the treatment of COPD disease, but elderly COPD patients have poor tolerance to surgery and a high probability of postoperative complications, which has seriously affected the postoperative recovery and quality of life of patients [8].

Studies have confirmed that when elderly COPD patients undergo surgical treatment, factors such as the patient's pulmonary function, surgical stimulation, and residual anesthetics will cause the patient's airway pressure to increase during the operation, which will lead to difficulty in postoperative extubation and hypoxemia, bronchospasm, and cardiovascular instability thus seriously affecting the patient's respiratory function and postoperative recovery effect [9, 10]. Thoracic and upper abdominal surgery can lead to secondary respiratory complications in COPD patients, and the risk is high. Therefore, it is very important to choose anesthesia methods for patients. GA combined with SA is regarded as a very effective perioperative management method for high-risk patients with large surgical trauma [11]. Studies have confirmed that GA combined with SA is more effective than GA alone, and it is more suitable for thoracic and upper abdominal surgery in elderly patients [12, 13].

RETRACTED

This work compared the effects of simple GA and GA+SA on various indicators such as anesthesia and anesthesia recovery, postoperative analgesia, and cognitive function in elderly patients with COPD. This work is aimed at providing a reference for improving the anesthesia effect of elderly patients with COPD surgery, improving the success rate of surgery, reducing the incidence of postoperative respiratory events, and accelerating the postoperative recovery effect of patients.

The major contribution of this paper is given below:

- In this paper, the researchers have analyzed the efficacy and safety of general anesthesia (GA) combined with spinal anesthesia (SA) (GA+SA) in elderly patients with chronic obstructive pulmonary disease (COPD)
- A total of 50 patients admitted to the hospital were divided into two groups: the control group and the observational group
- The control group was treated with simple GA and the observational group with GA+SA
- The results of the comparison of basic data of patients, comparison of surgical conditions, comparison of breathing circulation indicators, comparison of BUN and Scr levels, comparison of analgesic effect, comparison of pulmonary function, comparison of inflammatory factor levels, comparison of cognitive function, and comparison of incidence of respiratory system events are assessed
- Research in this study showed that GA+SA can greatly increase the dosage of GA drugs, accelerate the recovery time of patients, and improve the quality of recovery and postoperative analgesia

The outline of this paper is given below.

In Section 2, Materials and Methods, the general information of the selected patients is collected. The methods used to treat the observational group and the control group are discussed. In Section 3, the results obtained from the control group and the experimental group are discussed. In Section 4, the causes and effects of patient suffering from COPD respiratory disease are discussed.

## 2. Materials and Methods

In this section, the general information of the selected patients is collected and divided into the control group (simple GA) and the observational group (GA+SA). The research methods for the treatment of patients are discussed. The observation index and statistical analysis are also discussed.

### 2.1. Research Subjects

50 patients with COPD who were treated in the Affiliated Hospital of Hebei Engineering University from March 2020 to December 2021 were enrolled as the research subjects. They had to meet the below criteria.

RETRACTED

Inclusion criteria: patients whose diagnosis was in line with the clinical diagnostic criteria for COPD formulated by the Third China Pulmonary Heart Disease Conference in 1983 and patients who did not receive any immunosuppressive or hormone therapy before surgery.

Exclusion criteria: patients with consumptive diseases such as cardiovascular system diseases, endocrine system diseases, immune system diseases, inflammation, and malignant tumors; patients with abnormal liver and kidney function; and patients with hematological diseases.

Ethical approval: the experiment had been approved by the medical ethics committee of the Affiliated Hospital of Hebei Engineering University. All the included subjects were aware of the trial process and signed the informed consent.

### 2.2. Grouping and Treatment Methods of Subjects

The patients were rolled randomly into an observation group and a control group, with 25 cases in each group. The patients in the control group were treated with the GA method, and the patients in the observation group were treated with GA+SA. The methods of anesthesia for different groups of patients were as follows.

Patients in the control group were treated with a simple GA method, and their vital signs were routinely monitored. The patients were induced by intravenous injection of midazolam and propofol, respectively, to promote muscle relaxation and injected with rocuronium bromide injection. After the injection, the patients were intubated. The combined injections during anesthesia were propofol plus remifentanil and rocuronium bromide injection. The patient's various signs and data should be observed and the dose adjusted according to the patient's condition.

The patients in the observation group were treated with GA+SA. The specific operation method of GA was the same as that of the control group, and the operation was completed as above. Combined SA and epidural anesthesia were used, the puncture point was the L2-3 intervertebral space, and the spinal anesthesia medication was 0.5% bupivacaine hydrochloride 1 mL. The injection time was 30 s, and the adjustment plane was T after the supine position. The sensory level was left and right, and 3–5 mL of 2% lidocaine was given epidurally when the anesthesia level was insufficient. After the anesthesia plane was fixed, dexmedetomidine was continuously infused intravenously at an infusion rate of 0.4 *μ*g·kg·h. After 10 minutes, the infusion rate was reduced to 0.2–0.4 *μ*g·kg·h. The EEG bispectral index value was controlled at 75~85 as the standard.

RETRACTED

### 2.3. Observation Indicators

1. It should monitor the basic indicators: mean arterial pressure (MBP), heart rate (HR), blood oxygen saturation (SaO_2_), and blood oxygen concentration (PaO_2_) of patients before anesthesia (T0), at the time of skin incision (T1), and 1 hour after surgery (T2). 5 mL of venous blood was collected from the patients, and the blood glucose (BG), blood urea nitrogen (BUN), and serum creatinine (Scr) levels were measured
2. Surgery-related indicators: the operation time, PRT, LET, the number of anesthetic drugs (propofol, rocuronium, and fentanyl drugs), and CET were recorded
3. The postoperative pain intensity of patients was scored using the verbal rating scale (VRS) [14]. The VRS consisted of a series of adjectives used to describe pain, and the descriptors were arranged in order from the least to most painful. VRS covered a 4-level scoring method, a 5-level scoring method, and other methods. In this work, the 4-level scoring method was used to evaluate the postoperative pain intensity of patients
4. Pulmonary function indicators included forced vital capacity (FVC), forced expiratory volume in the first second/forced vital capacity (FEV1/FVC), and forced expiratory flow (FEF) 25%~75% in the next morning after surgery
5. Inflammatory indicators: venous blood was collected from patients before anesthesia (0 h), 1 h after surgery (1 h), and 1 d (24 h) after surgery. The enzyme-linked immunosorbent assay was used to detect interleukin-6 (IL-6), interleukin-8 (IL-8), and serum tumor necrosis factor-*α* (TNF-*α*) levels
6. Mental state evaluation: the SPMSQ was adopted to evaluate the recovery of the mental state of patients at 0 h before surgery, 1 h after surgery, 6 h after surgery, 12 h after surgery, and 24 h after surgery [15]. The scale included 10 evaluation dimensions including short-term and long-term memory, environmental perception, daily events, and computing ability. Evaluation criteria: 0~2 points for patients with complete cognitive function, 3~4 points for patients with mild cognitive impairment, 5~7 points for patients with moderate cognitive impairment, and 8~10 points for patients with severe cognitive impairment
7. EMG evoked potentials were applied to detect the P300 wave of ERPs in patients, and the sequence of “auditory target stimulation/nontarget stimulation” was selected to induce related event potentials. The patient was required to sit on a soft chair, relax the muscles of his body, close his eyes, and keep his mind clear and focused. The P3 latency and P3 amplitude under target stimulation were detected at 0 h before surgery, 1 h after surgery, 6 h after surgery, 12 h after surgery, and 24 h after surgery
8. The probability of respiratory system events was counted, including pulmonary infection, atelectasis, bronchospasm, bronchoscopy, and noninvasive positive pressure ventilation (NPPV) support

RETRACTED

### 2.4. Statistical Methods

SPSS 19.0 statistical software was adopted for data processing and analysis. Measurement data were expressed as mean ± standard deviation (mean ± SD), and independent samples *t*-test was used for analysis between groups. The count data were expressed by frequency (%), and the chi-square test was used for analysis between groups. *P* < 0.05 was considered to have a statistically significant difference.

## 3. Results

In this section, the results of the comparison of basic data of patients, comparison of surgical conditions, comparison of breathing circulation indicators, comparison of BUN and Scr levels, comparison of analgesic effect, comparison of pulmonary function, comparison of inflammatory factor levels, comparison of cognitive function, and comparison of incidence of respiratory system events are assessed.

### 3.1. Comparison of Basic Data of Patients

The differences in general data of patients in two groups were compared (the results are shown in Table 1). No great difference was found in the gender ratio, average age, average course of the disease, average body weight, proportion of thoracic surgery, and upper abdominal surgery of patients between the two groups (*P* > 0.05).

### 3.2. Comparison of Surgical Conditions

The differences in operation time, recovery time, LET, AD, and CET were compared, and the results are displayed in Figure 1. The operation time, recovery time, LET, AD, and CET of the control group were 177.34 ± 8.91 min, 53.39 ± 7.54 min, 69.03 ± 6.11 min, 2013.72 ± 155.42 mL, and 33.46 ± 8.97 min, respectively; while those in the observation group were 181.89 ± 7.79 min, 22.01 ± 5.38 min, 33.52 ± 3.79 min, 1672.19 ± 142.93 mL, and 12.88 ± 3.21 min, respectively.

Compared with the control group, the recovery time, LET, and CET of the patients in the observation group were greatly shortened, and the AD was reduced (*P* < 0.05).

### 3.3. Comparison of Breathing Circulation Indicators

The differences in the levels of respiratory circulation evaluation indicators (MAP and HR) were compared at different time points (Figure 2). The MAPs at T0, T1, and T2 in the control group were 81.18 ± 3.14 mmHg, 92.36 ± 3.55 mmHg, and 90.62 ± 5.09 mmHg, respectively; and the HRs were 96 ± 5 min, 73 ± 6 min, and 86 ± 6 min, respectively. The MAPs in the observation group were 80.03 ± 4.28 mmHg, 97.81 ± 4.33 mmHg, and 81.25 ± 5.05 mmHg, respectively; and the HRs were 95 ± 4 min, 78 ± 7 min, and 92 ± 6 min, respectively.

RETRACTED

Compared with T0, the control group at T1 and T2 and the observation group at T1 had significantly higher MAP levels and significantly lower HR levels (*P* < 0.05). Compared with the control group, the MAP level of the observation group at T2 was observably decreased, while the MAP and HR levels of the observation group at T1 and T2 were increased at T1 (*P* < 0.05).

The differences in the levels of SaO_2_ and PaO_2_ and the evaluation indexes of respiratory and circulation were compared at different time points (Figure 3). The SaO_2_ at T0, T1, and T2 in the control group were 68.92 ± 4.15 mmHg, 64.49 ± 5.09 mmHg, and 67.73 ± 5.18 mmHg, respectively, and the PaO_2_ were 75.09 ± 4.08%, 78.81 ± 4.16%, and 75.54 ± 3.39%, respectively. The SaO_2_ in the observation group were 69.14 ± 5.33 mmHg, 82.25 ± 4.89 mmHg, and 77.16 ± 4.02 mmHg, respectively; and the PaO_2_ were 73.32 ± 3.31%, 88.19 ± 5.11%, and 80.04 ± 5.72%, respectively.

Compared with time T0, no obvious difference was found in the levels of SaO_2_ and PaO_2_ in the control group at time T1 and T2 (*P* > 0.05), while the levels of each index in the observation group were significantly increased (*P* < 0.05). Compared with the controls, the levels of SaO_2_ and PaO_2_ in the observation group at T1 and T2 were greatly increased (*P* < 0.05).

### 3.4. Comparison of BUN and Scr Levels

The differences in BUN and Scr levels between the two groups at different time points were compared (as illustrated in Figure 4). The BUN levels at T0, T1, and T2 of controls were 90.11 ± 5.03 *μ*mol/L, 70.61 ± 6.11 *μ*mol/L, and 81.55 ± 5.78 *μ*mol/L, respectively; and the Scr levels were 8.43 ± 0.65 mmol/L, 5.07 ± 0.71 mmol/L, and 4.52 ± 0.48 mmol/L, respectively. The BUN levels in the observation group were 89.77 ± 5.16 mmHg, 53.56 ± 4.99 *μ*mol/L, and 63.41 ± 4.26 *μ*mol/L, and the Scr levels were 8.55 ± 0.32 mmol/L, 6.67 ± 0.41 mmol/L, and 5.03 ± 0.46 mmol/L, respectively.

Compared with T0, the BUN and Scr levels of the control group and the observation group were sharply decreased at T1 and T2 (*P* < 0.05). Compared with the control group, the level of BUN in the observation group at T1 and T2 was decreased, and the level of Scr was increased (*P* < 0.05).

### 3.5. Comparison of Analgesic Effect

The differences in postoperative pain VRS scores of patients who received simple GA and GA+SA at different time points were compared (Figure 5). At 6 h, 12 h, 24 h, and 48 h after surgery, the number of cases with a VRS score less than 1 in the observation group was less than that in the control group, showing statistically obvious differences (*P* < 0.05).

### 3.6. Comparison of Pulmonary Function

The differences in the pulmonary function indicators of the patients were compared before and after surgery (Figure 6). Before surgery, the levels of FVC, FEV1/FVC, and FEF25%~75% for patients who received GA only and GA+SA were 2219.3 ± 209.2 mL vs. 2304.5 ± 211.6 mL, 56.71 ± 2.33% vs. 57.09 ± 4.08%, and 0.75 ± 0.11 L/s vs. 0.77 ± 0.08 L/s, respectively, showing no observable differences (*P* > 0.05). After surgery, the above three indicators in the control and observation groups were 829.9 ± 189.3 mL vs. 1299.8 ± 201.5 mL, 35.88 ± 4.17% vs. 47.03 ± 4.21%, and 0.36 ± 0.09 L/s vs. 0.55 ± 0.10 L/s, respectively.

RETRACTED

Compared with before surgery, the levels of FVC, FEV1/FVC, and FEF25%-75% in the control and observation groups were notably decreased (*P* < 0.05). The postoperative levels of FVC, FEV1/FVC, and FEF25%-75% in the observation group were increased (*P* < 0.05).

### 3.7. Comparison of Inflammatory Factor Levels

The differences in the levels of serum inflammatory factors were compared between different groups at different time points (Figure 7). The IL-6 levels were 12.95 ± 1.14 pg/mL, 10.51 ± 1.02 pg/mL, and 9.61 ± 0.97 pg/mL before surgery and 1 h and 24 h after the surgery, respectively; the IL-8 levels were 11.03 ± 0.66 pg/mL, 10.12 ± 0.98 pg/mL, and 9.03 ± 0.55 pg/mL, respectively, at the above three time points; and the levels of TNF-*α* were 13.61 ± 1.03 pg/mL, 11.56 ± 0.88 pg/mL, and 10.23 ± 0.91 pg/mL, respectively. The IL-6 levels at each time point in the observation group were 12.88 ± 1.23 pg/mL, 9.63 ± 1.09 pg/mL, and 7.79 ± 0.88 pg/mL, respectively; IL-6 levels were 10.97 ± 0.87 pg/mL, 9.11 ± 0.91 pg/mL, and 6.53 ± 0.62 pg/mL, respectively; and the TNF-*α* levels were 13.55 ± 0.92 pg/mL, 10.39 ± 0.86 pg/mL, and 8.71 ± 0.65 pg/mL, respectively.

It indicated that compared with T0, the levels of IL-6, IL-8, and TNF-*α* in both groups were greatly decreased at T1 and T2 (*P* < 0.05); and they in the observation group at T1 and T2 were decreased (*P* < 0.05).

### 3.8. Comparison of Cognitive Function

The differences in SPMSQ scores at different time points were compared (Figure 8). It was 1.98 ± 0.21 points, 1.67 ± 0.22 points, 1.54 ± 0.14 points, 1.22 ± 0.10 points, and 1.16 ± 0.08 points at different time points for patients that received simple GA. The scores at each time point were 2.03 ± 0.16, 1.70 ± 0.21, 1.15 ± 0.16, 0.66 ± 0.09, and 0.23 ± 0.05, respectively, for patients that received GA+SA.

Compared with preoperative 0 h, the SPMSQ scores of all patients were decreased at 1 h, 6 h, 12 h, and 24 h after the surgery (*P* < 0.05). In contrast to the scores of patients who received simple GA, the SPMSQ scores of those who received GA+SA were decreased at 6 h, 12 h, and 24 h after surgery (*P* < 0.05).

RETRACTED

The differences in EMG P3 latency and amplitude were compared at different time points (Figure 9). The P3 latency of patients who received GA was 301.3 ± 10.9, 414.7 ± 11.3, 390.5 ± 12.5, 361.2 ± 14.1, and 355.4 ± 14.6 at 0 h, 1 h, 6 h, 12 h, and 24 h after the surgery, respectively; while the P3 amplitudes were 14.1 ± 1.2, 6.2 ± 1.4, 10.1 ± 0.9, 11.6 ± 1.0, and 13.3 ± 1.1, respectively. The P3 latency at each time point for patients who received GA+SA was 298.7 ± 13.8, 356.9 ± 14.2, 320.8 ± 11.8, 288.4 ± 12.6, and 280.1 ± 14.1, respectively; while the P3 amplitudes were 14.0 ± 0.8, 9.5 ± 0.9, 11.8 ± 1.1, 13.0 ± 1.0, and 13.9 ± 0.8, respectively.

In both groups, the P3 latency period reached a peak at 1 h after the surgery, while the P3 waveform reached the minimum. Compared with 0 h before surgery, the P3 latency of the control group was significantly prolonged at 1 h, 6 h, 12 h, and 24 h after surgery, while the P3 amplitude was decreased (*P* < 0.05). Compared with preoperative 0 h, the P3 latency of the observation group was significantly prolonged at postoperative 1 h and 6 h, while the P3 amplitude was remarkably reduced (*P* < 0.05). Compared with the control group, the P3 latency in the observation group was shortened at postoperative 1 h, 6 h, 12 h, and 24 h, and the P3 amplitude was increased (*P* < 0.05).

### 3.9. Comparison of Incidence of Respiratory System Events

The differences in postoperative respiratory events (including pulmonary infection, atelectasis, bronchospasm, bronchoscopy, and NPPV support) were compared between both groups (Figure 10). In the control group, there were 4 cases (16%) of pulmonary infection, 2 cases (8%) of atelectasis, 7 cases (28%) of bronchospasm, 6 cases (24%) of bronchoscopy, and 4 cases of NPPV support (16%). In the observation group, there was 1 case (4%) of pulmonary infection, 0 case of atelectasis (0%), 3 cases of bronchospasm (12%), 0 case of sputum suction by fiberoptic bronchoscope (0%), and 0 cases of NPPV support (0%). The probability of postoperative respiratory system events in patients who received GA+SA was significantly lower than that in the control group (*P* < 0.05).

## 4. Discussion

COPD is a class of respiratory diseases characterized by airway airflow limitation that is irreversible and progressive [16]. High airway response can cause severe bronchospasm in COPD patients when they are exposed to adverse stimuli. During surgery, elderly COPD patients will be stimulated by anesthesia, intubation, extubation, and surgery, which affect the normal respiratory function of patients and increase the risk of surgery [17]. Appropriate postoperative analgesia can improve the efficacy and safety of surgical treatment. GA+SA can effectively inhibit the stress response of patients due to surgical trauma, improve the patient's metabolism, and reduce the use of anesthetic drugs [18]. Studies have confirmed that effective postoperative analgesia such as GA+SA can block the pain transmission of the central nervous system by inhibiting neuronal excitation in the surgical area. This can reduce the incidence of postoperative adverse reactions in patients and have a positive impact on the surgical treatment effect of patients [19, 20]. To this end, this work analyzed the use of GA combined with SA in the surgical treatment of elderly patients with COPD and evaluated the efficacy and safety of anesthesia.

RETRACTED

Due to the reduced physical function of elderly COPD patients, the use of anesthetic drugs has a more pronounced impact on elderly patients [21]. SA refers to the injection of drugs into the spinal cavity of the patient to block the nerve conduction function to achieve the purpose of anesthesia. The amount of anesthetic drugs used in SA is less, which is beneficial to the postoperative recovery of the patient [22, 23]. The results of this work showed that compared with GA alone, GA+SA patients significantly reduced the number of anesthetics used, recovery time, LET, and CET, which was consistent with the results of Ehsani et al. [24]. Then, this work adopted MAP, HR, SaO_2_, and PaO_2_ to evaluate the respiratory function of patients. The results showed that compared with simple GA, the postoperative MAP, SaO_2_, and PaO_2_ levels in patients with GA+SA were increased, while HR was similar to those before surgery. Secondly, this work evaluated the pulmonary function of elderly COPD patients under different anesthesia interventions by measuring FVC, FEV1/FVC, and FEF25%-75%. The results showed that the postoperative levels of FVC, FEV1/FVC, and FEF25%-75% in patients with GA+SA were much higher than those with GA alone. It is shown that GA+SA does not inhibit the respiratory and circulatory function of elderly patients with COPD surgery and does not affect the pulmonary function of patients [25].

Studies have confirmed that the secretion of cytokines and inflammatory mediators in COPD patients can cause damage to the alveoli and damage the airway wall structure of patients [26]. Elevated inflammatory factors can affect the generation and release of intracellular oxygen free radicals, thereby causing damage to lung tissue and cells in the airways, reducing pulmonary function in patients, and causing alveolar damage and airway remodeling [27, 28]. To this end, the changes in the levels of cytokines and inflammatory factors in the perioperative period of the two groups of patients were evaluated. The results showed that the postoperative serum levels in patients with GA+SA were lower than those of GA alone, and the postoperative analgesia VRS score was better. It shows that GA+SA can effectively reduce the levels of cells and inflammatory factors in elderly patients with COPD surgery and improve the anesthesia and analgesic effects of patients. The SPMSQ scale is a tool for evaluating the cognitive function status of patients, which can reflect the mental state and cognitive function of patients [29]. The results of this work showed that the postoperative SPMSQ score in patients with GA+SA was lower than that in patients with GA alone. Because the GA method requires the use of a large number of anesthetics to block neuronal signaling and also reduces the patient's cerebral blood flow, it will cause postoperative cognitive impairment in patients [30, 31]. In contrast, SA uses a small number of anesthetics and injects anesthesia into the spinal canal space to block neurons. For this reason, the degree of damage to the cognitive function of the patient is low, and the postoperative cognitive function of the patient can be improved [21, 32, 33]. Finally, this work compared the differences in the probability of postoperative respiratory events among patients. The results revealed that the incidence of postoperative pulmonary infection, atelectasis, bronchospasm, bronchoscopy, and NPPV support in patients with GA+SA was greatly lower than that in patients with GA alone. This is because GA+SA uses a small number of anesthetics, which improves the analgesic quality of patients so that patients have no obvious pain when coughing. This in turn guarantees the patient's treatment and restores confidence and ultimately reduces the incidence of pulmonary complications.

RETRACTED

## 5. Conclusions

This work is aimed at comparing the efficacy and safety of GA alone and GA+SA in elderly patients with COPD surgery. It was confirmed that GA+SA can greatly increase the dosage of GA drugs, accelerate the recovery time of patients, and improve the quality of recovery and postoperative analgesia. At the same time, GA+SA can also improve the respiratory function and cognitive function impairment of patients and reduce the level of postoperative inflammatory factors and the incidence of pulmonary complications, which is beneficial to the recovery of patients after surgery. However, this work only analyzed the effect of GA+SA on the short-term efficacy of elderly patients with COPD surgery and did not consider its impact on the patient's immune function and long-term prognosis. In future studies, it would focus on conducting in-depth follow-up studies in this research direction. In conclusion, the results of this work could provide a reference for the clinical application of GA+SA in elderly patients with COPD surgery.

## Figures and Tables

**Figure 1:** Comparison of surgery-related indicators. ∗ meant *P* < 0.05.

**Figure 2:** Changes in MAP and HR during the perioperative period. ∗, #, and & indicated *P* < 0.05 compared with the value of the control group at T0, the value of the observation group at T0, and the value of control at the same time point, respectively.

**Figure 3:** Changes in SaO_2_ and PaO_2_ during the perioperative period. # and & suggested *P* < 0.05 in contrast to the value of the observation group at T0 and the value of the control group at the same time point, respectively.

**Figure 4:** Changes in BUN and Scr during the perioperative period. ∗, #, and & indicated *P* < 0.05 compared with the value of the control group at T0, the value of the observation group at T0, and the value of control at the same time point, respectively.

**Figure 5:** The proportion of VRS pain scores.

**Figure 6:** Changes in pulmonary function indicators. ∗ and # indicated *P* < 0.05 in contrast to the controls before and after the surgery, respectively.

**Figure 7:** Changes in serum inflammatory factors during the perioperative period. ∗, #, and & suggested *P* < 0.05 compared to the value in the control group and the observation group before the surgery and the value of the control group after the surgery, respectively.

**Figure 8:** Comparison of SPMSQ score during the perioperative period. ∗, #, and & indicated *P* < 0.05 in contrast to the scores before the surgery in the control and observation groups and the score of the control group at the same time point, respectively.

**Figure 9:** Changes in P3 latency and amplitude of EMG signal during the perioperative period. ∗, #, and & meant *P* < 0.05 to the value in the control and observation groups before surgery and that in the control group at the same time point, respectively.

**Figure 10:** Comparison of postoperative respiratory system events. I~V referred to pulmonary infection, atelectasis, bronchospasm, bronchoscopy, and NPPV support, respectively.

**Table 1:** Comparison of basic data of patients.

Item	Control group	Observation group	*P* value
Sample size	25	25	
Male [*n* (%)]	19 (76)	20 (80)	0.665
Age (years old)	68.1 ± 2.7	69.0 ± 3.3	0.518
Disease duration (years)	3.5 ± 0.4	3.4 ± 0.3	0.434
Weight (kg)	62.7 ± 5.1	63.3 ± 4.9	0.509
Thoracic surgery [*n* (%)]	14 (56)	12 (48)	0.612
Upper abdominal surgery [*n* (%)]	11 (44)	13 (52)	0.433

RETRACTED

## Data Availability

The datasets used during the current study are available from the corresponding author on reasonable request.
